# Impact of Alendronate Sodium plus Elcatonin on Postoperative Bone Pain in Patients with Osteoporotic Fractures

**DOI:** 10.1155/2022/1213278

**Published:** 2022-09-07

**Authors:** Baohui Wang, Yindi Sun, Da Shi, Xiuwei Han, Na Liu, Bo Wang

**Affiliations:** ^1^Pain Ward of Orthopedics Department of TCM, Honghui Hospital, Xi'an Jiaotong University, Xi'an, 710000 Shaanxi Province, China; ^2^Joint Ward of Orthopedics Department of TCM, Honghui Hospital, Xi'an Jiaotong University, Xi'an, 710000 Shaanxi Province, China

## Abstract

**Objective:**

This research aims to investigate and analyze the impact of alendronate sodium (ALN) plus elcatonin (EC) in treating postoperative bone pain (BP) in patients with osteoporotic fractures (OPFs).

**Methods:**

One hundred and thirty-eight cases of OPFs admitted between July 2018 and July 2021 were selected, of which 68 cases receiving ALN were set as the control group and 70 cases receiving ALN plus EC were set as the research group. Intercomparisons were performed in terms of BP, curative effect, complication rate, and serum bone metabolism indexes such as bone Gla protein (BGP), parathyroid hormone (PTH), and bone alkaline phosphatase (BALP).

**Results:**

Better postoperative BP relief, higher overall response rate, and lower complication rate were identified in the research group versus the control group. On the other hand, the research group presented with increased BGP and BALP after treatment, higher than those in the control group, while the posttreament PTH decreased obviously and was lower versus the control group.

**Conclusions:**

For OPF patients, ALN plus EC contributes to significantly reduced postoperative BP, improved clinical efficacy, higher treatment safety, and better bone metabolism, which has high clinical application value.

## 1. Introduction

Osteoporosis (OP), one of the most prevalent systemic metabolic bone conditions, is mainly characterized by decreased bone mineral density and bone mass as well as abnormal bone microstructure, resulting in increased bone fragility and consequently elevated risk of fractures [1, 2]. As indicated by related statistics, the number of global OP patients has exceeded 200 million, with approximately 9 million new cases and as many as 1.5 million osteoporotic fracture (OPF) patients in the United States each year [3]. OPFs, which account for about 80% of all fractures, are usually caused by injury or bone lesion-induced stress [4, 5]. OPFs are shown to be often accompanied by postoperative bone pain (BP), which adversely affects patients' physical and mental health as well as activities of daily living [6]. Moreover, if OPFs are not timely intervened and alleviated, they are prone to refractures, further increasing the risk of disability in patients [7]. Further research on the treatment and intervention of OPFs is therefore critical for management optimization of such patients and reducing the incidence of OPF-related morbidity and disability rates.

At present, the treatment of OPFs is challenging, with a high risk of postoperative complications. Postoperative drug therapy is helpful to improve bone metabolism balance and relieve postoperative BP [8, 9]. Of them, alendronate sodium (ALN) is a commonly used oral bisphosphonate for the treatment of OP, which can prevent brittle fractures by promoting osteoclast (OC) apoptosis and preventing bone resorption [10]. In addition, it can help reduce the overall fracture risk in OP patients, providing long-term benefits for women with extremely high clinical vertebral fracture risk [11]. Reported by Deardorff et al. [12], ALN was preventive against nonvertebral fractures in postmenopausal OP women. Elcatonin (EC), which is also an antibone resorption drug like ALN, mainly inhibits bone resorption by reducing the number of OCs and inhibiting their secretory activity [13]. Animal experiments show that EC can inhibit the systemic acceleration of bone resorption and bone turnover caused by bone injuries without delaying the healing process of bone defects, which has a good effect on fracture healing [14]. EC has also been shown to help patients with osteoporotic vertebral fractures relieve pain, inhibit bone resorption, and improve their quality of life [15]. Another study has pointed out that EC can be combined with ALN to act on ovaries removed rats, which has a synergistic enhancement effect on trabecular structure and bone strength of mice [16].

Given the current lack of related research on ALN plus EC in relieving postoperative BP in OPF patients, this study aims to fill the gap and provide new insights into OPF treatment.

## 2. Materials and Methods

### 2.1. Baseline Information

From July 2018 to July 2021, 138 patients with OPFs were selected, with 68 patients receiving ALN and the other 70 patients treated with ALN plus EC being assigned to control group and research group, respectively. The control group had 26 males and 42 females aged 62.89 ± 5.65 years on average, and the disease course was 4.21 ± 1.04 years; the research group had 25 males and 45 females, with a mean age and a course of disease of (62.68 ± 9.24) years and (4.43 ± 1.47) years, respectively. The two groups showed comparable baseline information (*P* > 0.05). This study, carried out in strict compliance with the Declaration of Helsinki, has obtained approval from the Ethics Committee of Honghui Hospital, Xi'an Jiaotong University, as well as informed consent from all participants.

### 2.2. Eligibility Criteria

All patients enrolled were confirmed with primary OP and fractures caused by it, with surgical treatment, postoperative BP, and no other recent treatment.

In contrast, those with fractures injured to spinal cord and nerve root, hyperthyroidism, malignant tumor, deterioration of organ function, and abnormal cognitive function or communication function were excluded, as well as those with allergies to the study medication. In addition, patients complicated by impairment, serious cardiovascular diseases, and those who did not take the medication as required were ruled out.

### 2.3. Therapies

Both cohorts were given oral calcium carbonate D3 600mg once a day and active vitamin D3 (0.25 *μ*g/time) twice daily after surgery. On this basis, the control group received ALN tablets (Beijing Fuyuan Pharmaceutical Co., Ltd., H20059029), per os, 70 mg/time, once a week. The research group was treated with EC injection (Luye Pharma Group, H20040338) by intramuscular injection on the basis of the control group, 10 U/time, twice a week. Patients in both groups were treated for half a year.

### 2.4. Endpoints

#### 2.4.1. BP

The severity of BP was assessed preoperatively and six months after treatment using the Visual Analogue Scale (VAS) [17], an instrument with a score range of 0-10 points and the score in direct proportion to BP severity.

#### 2.4.2. Efficacy

Markedly effective was indicated if the fracture basically recovered after treatment, with normal shape, significantly increased bone mineral density, and basically disappeared pain; if patients showed fracture healing, with a certain degree of pain relief and increase in bone mineral density, it is considered effective; ineffective was considered if patients had no significant changes before and after treatment. The percentage of the sum of the cases with markedly effective and effective treatment in the total number of cases is the overall effective rate.

#### 2.4.3. Safety

The cases of gastrointestinal reactions, fever, headache, fatigue, and other complications were recorded, and the complication rate was calculated.

#### 2.4.4. Bone Metabolism

Bone metabolism was evaluated before and 6 months after intervention by detecting serum parameters such as bone Gla protein (BGP), bone alkaline phosphatase (BALP), and parathyroid hormone (PTH). Before the test, fasting cubital venous blood (5 mL) was sampled early in the morning. After serum separation, BGP, BALP, and PTH were detected by the enzyme-linked immunosorbent assay (ELISA), with the reagents all supplied by the Shanghai Fuyu Biotech.

### 2.5. Statistical Processing

Data analysis and picture drawing were carried out through the GraphPad Prism 6 (GraphPad Software, San Diego, USA). A chi-square test was used for intergroup comparison of count data recorded as case number/percentage (*n*/%). Mean ± SEM was used for measurement data, and the inter- and intragroup differences were identified by independent sample *t*-test and paired *t*-test, respectively. *P* < 0.05 was the significance level in this study.

## 3. Results

### 3.1. Baseline Data

The two cohorts of patients differed insignificantly in baseline data like sex, age, average age, disease course, etiology, fracture site, diabetes mellitus, hypertension, drinking/smoking history, and marital status (*P* > 0.05) (Table 1).

### 3.2. Postoperative BP in Two Groups

We evaluated patients' postoperative BP by the VAS. The two groups had no statistical difference in the pretreatment VAS score (*P* > 0.05). After treatment, the score reduced markedly in both cohorts (*P* < 0.05) and was lower in research group (*P* < 0.05) (Figure 1).

### 3.3. Clinical Efficacy of Two Groups

We analyzed the efficacy of the two groups to evaluate the impacts of the two interventions on patients' clinical outcomes. A statistically higher overall response rate was determined in research group when compared to control group (90.00% *vs.* 64.71%, *P* < 0.001) (Table 2).

### 3.4. Complication Rate of Two Groups

We observed and recorded the cases of gastrointestinal reactions, fever, headache, and fatigue and found no statistical difference in the complication rate between groups (*P* > 0.05) (Table 3).

### 3.5. Serum Bone Metabolism in Two Groups

By detecting BGP, BALP, and PTH, the impacts of the two interventions on patients' bone metabolism were evaluated. The three bone metabolism indices were not statistically different between them prior to treatment (*P* > 0.05). After intervention, BGP and BALP increased, while PTH decreased in both cohorts (*P* < 0.05), with higher BGP and BALP and lower PTH in research group as compared to control group (*P* < 0.05) (Figure 2).

## 4. Discussion

OP has a predilection for the elderly and women, and its pathological feature is the disequilibrium between bone formation and bone resorption [18]. The incidence of OPFs is constantly on the rise, and by 2025, there will be 3 million new OPF patients worldwide, bringing a huge economic burden to the healthcare system [19]. Moreover, such brittle fractures are linked to premature death and disability, which calls for related drug prevention [20]. Anti-OP drug intervention can help osteoporotic patients reduce the risk of fractures and complications [21].

ALN, as a first-line therapy, can validly lower the possibility of developing vertebral and nonvertebral fractures by inhibiting bone turnover and increasing bone mass, with a significant effect on improving bone strength [22]. ALN exerts an inhibitory effect on bone resorption through the mevalonate pathway, but it has to bind to plasma proteins due to low bioavailability, resulting in low bone tissue resorption rate and thus affecting the therapeutic effect [23]. EC is a derivative of eel calcitonin, which is synthesized by substituting disulfide bonds with vinyl bonds, with potent analgesic actions [24, 25]. Previous studies have confirmed that EC can be combined with bisphosphonates (such as risedronate) to treat patients with chronic back pain, with a pain-relieving effect [26]. In our study, 138 patients with OPFs were included, with the control group receiving ALN and the research group receiving ALN plus EC. The research group had a VAS score significantly lower than the pretreatment level and control group three months after therapy, suggesting that ALN plus EC can greatly reduce postoperative BP, with better pain relief efficacy than ALN alone. The analgesic effect of EC has also been verified in the rat neuropathic pain model, which can play an analgesic role by reversing the Na + channel abnormality induced by nerve injury [27]. In our research, the research group showed an obviously higher overall response rate while a similar complication rate than the control group, demonstrating that the combined therapy can improve patients' clinical outcomes and promote bone healing without increasing the incidence of adverse reactions.

Furthermore, we measured bone metabolism indexes to assess the influence of the two medication methods on bone metabolism of OPF patients. BGP and BALP are related indexes of bone formation. In the process of fracture healing, it is necessary to strengthen the bone formation function of osteoblasts, so as to regulate bone formation and promote bone healing [28]. PTH, a marker of bone turnover, can promote the release of bone calcium and phosphorus into blood by activating OCs, thus strengthening bone resorption and reducing bone mass [29]. As such, the increase of BGP and BALP levels and the decrease of PTH can help improve bone metabolism and inhibit acute bone loss, thus relieving OPF-associated BP to a certain extent [30]. In our research, the research group showed statistically higher posttreatment BGP and BALP and lower PTH than the pretreatment levels and control group, demonstrating far superior effects of the combined drug intervention on improving bone metabolism balance when compared to ALN monotherapy. EC is also shown to play an antibone resorption role by enhancing the osteoinduction related to recombinant human bone morphogenetic protein-2 and can promote the anabolism of osteoblasts [31]. According to Ji et al. [32], EC can inhibit bone resorption by binding to EC-like receptors on OC membrane, thus disrupting OC activity. Our study confirmed that patients with OPFs can relieve postoperative BP through the intervention of ALN plus EC, which provides a new idea for clinical management of such patients.

This study still shows room for improvement. First, the clinical sample size is small, which may have certain influence on the experimental results. Second, there is a lack of short-term and long-term prognosis analysis. If relevant analysis can be supplemented, it will help to further understand the impacts of the two intervention methods on the prognosis of OPF patients. Third, no relevant basic experiments have been carried out to reveal the mechanism of ALN combined with EC in the treatment of OPFs.

## 5. Conclusion

In summary, ALN plus EC can significantly reduce postoperative BP in patients with OPFs, improve curative efficacy, and enhance specific bone metabolism balance, with high safety and clinical promotion value.

## Figures and Tables

**Figure 1:** Postoperative bone pain. ^∗∗^*P* < 0.01.

**Figure 2:** Serum bone metabolism indexes. (a) BGP. (b) BALP. (c) PTH. Note: ^∗∗^*P* < 0.01.

**Table 1:** Patients' baseline data [*n* (%), mean ± SD].

Variables	*n*	Control group (*n* = 68)	Research group (*n* = 70)	*χ* ^2^/*t*	*P*
Sex				0.094	0.759
Male	51	26 (38.24)	25 (35.71)		
Female	87	42 (61.76)	45 (64.29)		
Age (years old)				1.289	0.256
<60	47	20 (29.41)	27 (38.57)		
≥60	91	48 (70.59)	43 (61.43)		
Average age (years)	138	62.89 ± 5.65	62.68 ± 9.24	0.161	0.873
Course of disease (years)	138	4.21 ± 1.04	4.43 ± 1.47	1.012	0.313
Etiology				0.294	0.863
Falls	79	38 (55.88)	41 (58.57)		
Collision	37	18 (26.47)	19 (27.14)		
Other accidents	22	12 (17.65)	10 (14.29)		
Fracture site				0.697	0.404
Intertrochanteric fracture of femur	80	37 (54.41)	43 (61.43)		
Femoral neck fracture	58	31 (45.59)	27 (38.57)		
Diabetes mellitus				0.264	0.608
No	68	32 (47.06)	36 (51.43)		
Yes	70	36 (52.94)	34 (48.57)		
Hypertension				1.450	0.229
No	46	26 (38.24)	20 (28.57)		
Yes	92	42 (61.76)	50 (71.43)		
Drinking history				0.452	0.501
No	65	34 (50.00)	31 (44.29)		
Yes	73	34 (50.00)	39 (55.71)		
Smoking history				0.014	0.907
No	44	22 (32.35)	22 (31.43)		
Yes	94	46 (67.65)	48 (68.57)		
Marital status				2.046	0.153
Single	39	23 (33.82)	16 (22.86)		
Married	99	45 (66.18)	54 (77.14)		

**Table 2:** Clinical efficacy of patients [*n* (%)].

Groups	*n*	Markedly effective	Effective	Ineffective	Total effective rate
Control group	68	19 (27.94)	25 (36.76)	24 (35.29)	44 (64.71)
Observation group	70	42 (60.00)	21 (30.00)	7 (10.00)	63 (90.00)
*χ* ^2^ value	—	—	—	—	12.670
*P* value	—	—	—	—	<0.001

**Table 3:** Complication rate of patients [*n* (%)].

Categories	Control group (*n* = 68)	Research group (*n* = 70)	*χ* ^2^ value	*P* value
Gastrointestinal reactions	5 (7.35)	7 (10.00)	—	—
Fever	0 (0.00)	2 (2.86)	—	—
Headache	2 (2.94)	0 (0.00)	—	—
Fatigue	0 (0.00)	1 (1.43)	—	—
Total incidence	7 (10.29)	10 (14.29)	0.509	0.476

## Data Availability

The labeled dataset used to support the findings of this study are available from the corresponding author upon request.
